# A Comparative Study of Four Total Variational Regularization Reconstruction Algorithms for Sparse-View Photoacoustic Imaging

**DOI:** 10.1155/2021/6622255

**Published:** 2021-10-18

**Authors:** Xueyan Liu, Limei Zhang, Yining Zhang, Lishan Qiao

**Affiliations:** Department of Mathematics Science, Liaocheng University, Shandong 252000, China

## Abstract

Photoacoustic imaging (PAI) is a new nonionizing, noninvasive biomedical imaging technology that has been employed to reconstruct the light absorption characteristics of biological tissues. The latest developments in compressed sensing (CS) technology have shown that it is possible to accurately reconstruct PAI images from sparse data, which can greatly reduce scanning time. This study focuses on the comparative analysis of different CS-based total variation regularization reconstruction algorithms, aimed at finding a method suitable for PAI image reconstruction. The performance of four total variation regularization algorithms is evaluated through the reconstruction experiment of sparse numerical simulation signal and agar phantom signal data. The evaluation parameters include the signal-to-noise ratio and normalized mean absolute error of the PAI image and the CPU time. The comparative results demonstrate that the TVAL3 algorithm can well balance the quality and efficiency of the reconstruction. The results of this study can provide some useful guidance for the development of the PAI sparse reconstruction algorithm.

## 1. Introduction

Photoacoustic imaging (PAI) is a novel noninvasive biomedical imaging modality with the capability of quantitatively imaging of light absorption characteristics of endogenous tissue chromophores that has grown tremendously in the last two decades [1–4]. As a hybrid imaging method, PAI combines strong optical contrast with high ultrasonic penetration [5–7]. And it has shown great potential in multiple clinical applications, including the breast imaging [8, 9], dermatologic imaging [10, 11], thyroid imaging [12, 13], and imaging of the lymphatic system [14]. In PAI, the reconstruction of a high-quality image usually requires a large amount of signal data, which requires expensive electronic equipment or long data acquisition times. Moreover, in many clinical applications including ophthalmic imaging [15] and breast imaging [8], only incomplete data with limited angles can be accepted. Additionally, the conventional analytic methods usually reconstruct distorted images with strong artifacts when the data are insufficient or collected from few views. Therefore, the development and investigation of high-speed and high-quality PAI image reconstruction algorithms based on incomplete data is a popular research area of current interest [16–18]. To address the issue of insufficient information, the iterative algorithms for PAI reconstruction have been proposed to improve the quality of reconstructed images and reduce the time of data acquisition [19–21]. The incomplete data may arise from a variety of forms, but in this work, we focus on the sparse data problem in PAI with a circular measurement geometry.

Mathematically, the reconstruction of PAI images from sparse data can be regarded as a problem of solving underdetermined linear equations. By incorporating some prior information of the object or missing data, the iterative algorithms that can obtain more accurate reconstruction results at the cost of much more computing time have been developed for PAI [19–21]. One of them is based on the theory of compressed sensing (CS), which has attracted more and more attention due to its can recover sparse signals using much less measurements than advised by Shannon's sampling theory [22, 23]. By using the L1magic convex optimization algorithm and sparse-view data, Provost and Lesage applied the CS theory to the PAI imaging for the first time [24]. The issue of loss of resolution and artifacts in the case of insufficient measurements can be solved by using random lighting via the SPGL1 algorithm [25]. Based on a set of highly sparse representations of noise signals, Bayesian CS theory was used to obtain PAI images [26]. The results of phantom and in vivo experiments showed that the CS method can effectively reduce the undersampling artifacts through the nonlinear conjugate gradient descent algorithm [27, 28]. All these studies showed that the CS-based iterative reconstruction methods can significantly reduce the number of ultrasound transducers in the PAI imaging system and obtain high-quality reconstructed images with sparse data.

The total variation (TV) regularization and compressed sensing theory has a wide array of applications in biomedical imaging, for its good properties for preserving sharp edges and contours of objects. For example, a TV iterative shrinkage scheme is proposed to CS recovery of parallel MRI [29, 30]. Jia et al. developed the GPU-based cone-beam CT reconstruction algorithm using noisy and reduced projection data via TV [31]. Liu et al. investigated the application of sparse Bayesian learning framework and in electrical impedance tomography [32, 33]. This paper conducts a quantitative performance study on the application of CS-based TV regularization reconstruction algorithm in PAI. The total variation minimization by augmented Lagrangian and alternating direction algorithm (TVAL3) [34, 35], the generic log-barrier algorithm (L1magic) [24, 36], Nesterov's algorithm (NESTA) [37], and the two-step iterative shrinkage thresholding algorithm (TwIST) [38] are considered to solve the TV minimization problem. Based on sparsely sampled data, we evaluated the performance of the four reconstruction algorithms. Both the quality of the reconstructed images and the CPU runtime are investigated. The results of this study are expected to provide a suitable reconstruction algorithm for PAI that reduces the scanning time without reducing the quality of the reconstructed image.

The organization of this article is as follows.  Section 2 briefly reviews the methods used in the study, including the photoacoustic theory, reconstruction algorithms, and evaluation criteria. The results of a comparative experimental study and discussion are presented in Section 3. In the last part of this article, we got some conclusions based on the results of numerical experiments and simulation experiments.

## 2. Methods

### 2.1. Photoacoustic Theory

According to the theory of photoacoustic signal generation, the relationship between the ultrasonic pressure *p*(**r**, *t*) in a homogeneous medium and the absorption distribution *A*(**r**) obeys the following wave equation [1]:

(1) $$\begin{array}{c} \nabla^{2}p\left(r,t\right)-\frac{1}{c^{2}}\frac{\partial^{2}}{\partial t^{2}}p\left(r,t\right)=-\frac{\beta }{C_{p}}A\left(r\right)\frac{\partial \delta \left(t\right)}{\partial t}, \end{array}$$

where **r** denotes the pixel coordinate, *t* means the time, *c* is the sound velocity, *β* is the thermal coefficient of volume expansion, *C*_*p*_ is the specific heat, and *δ*(*t*) is a delta function. By using the Green function, wave equation (1) can be solved, providing the forward problem [9].

(2) $$\begin{array}{c} p\left(r_{0},t\right)=\frac{\beta }{4\pi C_{p}}∭\frac{A\left(r\right)}{\;|\;r-r_{0}\;|\;}\delta \left(t-\frac{\;|\;r-r_{0}\;|\;}{c}\right){\text{d}}^{3}r, \end{array}$$

where **r**_0_ is the position of the ultrasound transducer.

By taking the Fourier transform of equation (2) and denoting *k* = *ω*/*c*, where *ω* is the angular frequency, the forward problem in the temporal-frequency domain can be expressed as [24]

(3) $$\begin{array}{c} \bar{p}\left(r_{0},k\right)=\frac{-ik\beta }{4\pi C_{p}}∭A\left(r\right)\frac{\exp\left(ik\left|r_{0}-r\right|\right)}{c\left|r_{0}-r\right|}d^{3}r. \end{array}$$

During the experiment, we obtained the photoacoustic signal in the frequency domain by performing fast Fourier transform on the time domain signal. After discretisation, equation (3) can be represented as a linear equation:

(4) $$\begin{array}{c} Y=KX, \end{array}$$

where *Y* ∈ *R*^*M*^ denotes the vector for all pressure measurements in Fourier domain and *X* ∈ *R*^*N*^ denotes the vector for the unknown reconstruction image. However, we can only observe inaccurate measurements *Y* = *KX* + *ε*, where *ε* ∈ *R*^*M*^ denotes the modeling transducer noise. According to equation (3), the time-frequency domain measurement matrix can be written as

(5) $$\begin{array}{c} K_{\left(m,n\right)\left(i,j\right)}=-{ick}_{n}\frac{e^{{ik}_{n}\left|r_{m}-r_{ij}\right|}}{\left|r_{m}-r_{ij}\right|},m=1,2,\cdots ,p,n=1,2,\cdots ,q, \end{array}$$

where *r*_*m*_ represents the transducer position, *r*_*ij*_ indicates the coordinate of pixel, *p* is the transducer quantity, and *q* represents the number of sampling locations, respectively. The image reconstruction problem is to extract the absorption distribution *X* from the pressure data *Y*, which is usually ill-posed when there are fewer sampling points. Therefore, regularization techniques and prior information of the image are utilized to obtain a stable reconstruction process.

### 2.2. Total Variation Regularization

So far, a variety of CS reconstruction algorithm has been developed, such as the greedy iterative algorithm, total variation (TV), and Bayesian framework. Among them, TV regularization has great success in image reconstruction due to its capability of keeping edges and boundaries. The discrete form of the isotropic TV for a grayscale image is the sum of the *L*_2_ norm of the discrete gradient:

(6) $$\begin{array}{c} \text{TV}\left(X\right)=\overset{N}{\underset{i=1}{\sum }}{\left\|D_{i}X\right\|}_{2}=\overset{N}{\underset{i=1}{\sum }}\sqrt{\Delta_{i}^{h}X^{2}+\Delta_{i}^{v}X^{2}}, \end{array}$$

where *D*_*i*_*X* = (Δ_*i*_^*h*^*X*, Δ_*i*_^*v*^*X*)^*T*^ is the discrete gradient of the gray image *X* and Δ_*i*_^*h*^ and Δ_*i*_^*v*^ denote the horizontal and vertical difference operators. The existing literature indicated that TV-based CS algorithms can accurately reconstruct images from sparsely sampled data [34–38]. The *L*_2_ norm of *D*_*i*_*X* corresponds to the isotropic TV, or the *L*_1_ norm of *D*_*i*_*X* corresponds to the anisotropic TV. In the field of PAI, the TV minimization optimization algorithm can reconstruct excellent image from few view data [39–42]. The noiseless discrete TV regularization model can be written as

(7) $$\begin{array}{c} \underset{X}{\min}TV\left(X\right)\;s.t.\;KX=Y. \end{array}$$

For the reconstruction with noise signals, we can solve the Rudin-Osher-Fatemi model as an alternative

(8) $$\begin{array}{c} \underset{X}{\min}TV\left(X\right)+\frac{\lambda }{2}{\left\|KX-Y\right\|}_{2}^{2}. \end{array}$$

In this work, the TVAL3, L1magic, NESTA, and TwIST are considered to solve TV minimization problem (7) or (8). Comparative performance is assessed for both noiseless and noisy sparsely sampled data.

### 2.3. Evaluation Factors

Three quantitative parameters are used to evaluate the performance of these four reconstruction algorithms from a sparse data set: the CPU time, the signal-to-noise ratio (SNR), and the normalized mean absolute error (NMAE). The CPU time was used to estimate the efficiency of the algorithm, and the SNR was applied to evaluate the quality of the reconstructed image, and the NMAE was used to quantify the reconstruction error between the gray image and its reconstruction. The SNR is defined by

(9) $$\begin{array}{c} \text{SNR}\left(\overset{⌢}{X}\right)=10*\log_{10}\left(\frac{{\left\|X-\bar{X}\right\|}^{2}}{{\left\|X-\overset{⌢}{X}\right\|}^{2}}\right), \end{array}$$

where $\overset{⌢}{X}$ is the reconstruction and $\bar{X}$ is the mean intensity valve of *X*. The NMAE is defined as

(10) $$\begin{array}{c} \text{NMAE}\left(\overset{⌢}{X}\right)=\frac{\left\|X-\overset{⌢}{X}\right\|}{\left\|X\right\|}\times 100\%. \end{array}$$

## 3. Experiments and Results

In this article, we provide a simulation-based comparative performance study between these four TV regularization algorithms. The forward simulation and inverse reconstruction were conducted in 2D phantoms. The NCAT phantom and the blood vessel phantom are used in the comparisons to generate the photoacoustic signals. And the photoacoustic signals are generated by using equation (3).  Figure 1(a) shows the NCAT phantom, and Figure 1(b) shows the blood vessel phantom. The size of the phantom is 42 mm × 42 mm with a resolution of 128 × 128 pixels. During the simulation, the sound speed is 1500 m/s and the diameter of the circular scan is 60 mm. To simulate the response of the ultrasonic transducer, at every sampling location, 64 randomly chosen *k*_*n*_/2*πc*'s inside the [0.1, 32] MHz window were employed to define the frequency domain projection matrix **K**. By rescaling the phantom gray values to [0, 1], we acquired the frequency domain signals using the projection matrix.

The simulation experiments were carried out using MATLAB (MathWorks, Natick, MA) on a personal computer with an Intel core i7-4790 processor and 32 GB memory. The parameter ranges of the four algorithms are selected according to the literature 34 to 38, and the specific parameter values are manually adjusted. The same iteration stopping criteria ‖*X*^*k*+1^ − *X*^*k*^‖/‖*X*^*k*^‖ < 0.005 were used to be fair to compare the four algorithms. In the following section, the quality of the reconstructed images and quantitative comparisons are going to be discussed.

### 3.1. Sparse-View Reconstruction

The reconstructed images of the NCAT phantom using these four TV regularization algorithms and TV regularization model (7) from a set of the sparsely sampled signals, with 20, 30, and 40 positions, are shown in Figure 2. The first column displays the reconstructed images of the TVAL3 algorithm, and the second column show those of the L1magic algorithm. The third column is the reconstructed images of the NESTA algorithm, and the fourth column presents those of the TwIST algorithm. From Figure 2, it can be found that the image of the NCAT phantom has been reconstructed very well by the TVAL3 algorithm, even when the sampling number is reduced to 20. There are stripe and speckle noise in the image reconstructed by the L1magic algorithm, which affects the quality of the reconstruction. The image reconstructed by the NESTA algorithm is blurred, which affects the visual effect. Among the four algorithms, the TwIST algorithm performed the worst. Even if signals with 40-view angles are used, the TwIST algorithm still cannot obtain a better image. The TwIST algorithm still cannot obtain a better image under 40-view sampling circumstance. This experiment shows that the TVAL3 method is better than other three methods significantly in PAI image sparse reconstruction.

In order to better observe the differences between these four algorithms, we drew the pixel gray scales along the middle extraction lines of the reconstructed images. In Figure 3, the red dotted line and the black solid line are the pixel gray scales of the reconstructed image and the NCAT phantom, respectively. By observing the gray scales, we can get the similar conclusions mentioned above. Therefore, when these two evaluation factors are considered together, the TVAL3 algorithm achieves the best reconstruction performance, followed by the L1magic algorithm and the NESTA algorithm.

The quantitative evaluation parameters of the reconstructed images including the CPU time, the SNR, and the NMAE achieved by these four algorithms. From the CPU time in Table 1, we can know that there are large differences between the algorithm execution times: TwIST is about 1.3 times faster than NESTA, which itself can be roughly 2 times faster than TVAL3. And the L1magic algorithm has the longest running time. As the sampling number increases, the SNR data show an upward tendency and the NMAE values show a downward tendency. According to Table 1, we find that the TVAL3 algorithm provides the highest SNR value and the lowest NMAE value and the TwIST algorithm has the lowest SNR value and the highest NMAE value. NESTA and L1magic have the similar reconstruction performance. Considering the reconstruction efficiency and performance, the TVAL3 algorithm is the optimal algorithm for sparsely sampling PAI.

Figure 4 illustrates the reconstructed images of the blood vessel phantom using these four TV regularization algorithms from a set of the sparsely sampled signals, with 20, 30, and 40 positions. Therein, the first column to the fourth column show the reconstruction results of the TVAL3 algorithm, the L1magic algorithm, the NESTA algorithm, and the TwIST algorithm, respectively. From Figure 4, we can see that the blood vessel phantom has been well reconstructed when using the TVAL3 algorithm and 40 position signals. The image quality of the reconstruction is reduced when 30 position signals are used. And the quality of image reconstructed by using 20 position signals becomes very poor. However, the reconstructed images contain noises and blurs when using the other three algorithms and 40 position signals, and the quality of the reconstructed images is relatively poor when 30 and 20 position signals are used. This experiment fully proves that the TVAL3 method has the best reconstructed image quality.

The detail distinguish ability can also be seen from the pixel gray scales along the middle extraction lines of the reconstructed images (the red line in Figure 1(b)). As can be seen from Figure 5, the TVAL3 algorithm has the best image detail reconstruction capability. The reconstructed image with L1magic algorithm contains more interference noise. The details of the image reconstructed by the NESTA algorithm are blurred. And the TwIST algorithm has the worst image detail reconstruction ability. According to Figure 5, we can get the similar conclusion as the previous NCAT phantom experiment.

We record the CPU time for these four algorithms in each experiment of the blood vessel phantom, as shown in Table 2. The CPU time of the TwIST algorithm is approximately 2.2 times longer than the NESTA algorithm, which itself is about 2.6 times faster than TVAL3. And the CPU time reconstructed by the L1magic algorithm is the longest. According to the SNR in Table 2, we can see that the TVAL3 algorithm can obtain a SNR of 30 dB using signals from 30-views, while the SNRs of the reconstructed images of the other three algorithms are less than 30 dB using signals from 60-views. Similarly, the TVAL3 algorithm provides the lowest NMAE value.

Considering the results of these two simulation experiments, we can draw a useful conclusion that the quality of reconstructed image with the TVAL3 algorithm is better than the other three algorithms. The artifacts and blurs emerge in the other three algorithms reconstructed images, and the quality of images is severely affected indicating that these three methods are not suitable for sparse reconstruction. From the simulation results, we can conclude that the TVAL3 algorithm is more suitable for reconstructing photoacoustic images under sparse sampling conditions than the other three algorithms.

### 3.2. Robustness to the Noise

In the actual photoacoustic imaging process, the signal will be affected by Gaussian white noise from the system ultrasonic transducer and electronic devices. Therefore, it is very important for an algorithm to keep stable performance in the presence of noise. In order to analyze the robustness of those four methods, we added different levels of Gaussian noise to the signal. Results of noisy signal experiments are evaluated by SNR and NMAE.

In Figure 6, the SNR and the NMAE indexes are represented as a function of the number of data. A good algorithm has a larger SNR and a smaller NMAE. Figure 6 shows the trend diagram of the SNR and NMAE between the NCAT phantom and the reconstruction obtained from those four methods and TV regularization model (8). We remind that higher SNR and lower NMAE indicate superior image quality. It is clear that the TVAL3 algorithm outperform the other three algorithms also in terms of the SNR and NMAE. Moreover, the TVAL3 algorithm can not only obtain better performance with fewer measurements but also improve SNRs faster than the other three algorithms.

It can be seen from Figure 7, when there is weak noise of 40 dB and 30 dB, those four methods achieve similar SNRs and NMAEs when using signals with less than 25 positions. Furthermore, the TVAL3 algorithm achieves the biggest SNR and the smallest NMAE with sampling locations of more than 40 and improves SNR faster than the other three algorithms. When there is strong noise of 20 dB and 10 dB, the NESTA algorithm and the TwIST algorithm have smaller SNRs and larger NMAEs, but the TVAL3 algorithm can still achieve good reconstruction results with sufficient measurements. In other words, the TVAL3 algorithm achieves good reconstruction of PAI images in noisy environments.

Figure 8 shows the histogram of the influence of changing variance of Gaussian noise distribution on TVAL3. When the number of signals is small, there is not a great deal of difference in the SNR of reconstructed images with different levels of noise signals. While the number of signals exceeds 25, the SNR of the reconstructed images under different noise levels will vary greatly. It can also be seen from Figure 8 that the SNR of the reconstructed image can be improved by increasing the number of signals when the noise level is low, and the SNR of the reconstructed image is low when the noise level is high. Therefore, the biggest challenge in practical experiments is how to minimize the impact of noise. Signal averaging technology is needed to eliminate noise interference and obtain more reliable and effective signal data.

### 3.3. In Vitro Experiments

We also compared those four reconstruction algorithms through in vitro experiment.  Figure 9(a) shows the schematic diagram of the circular scanning experimental system, which is modified from our previous article. A Q-switched 532 nm Nd : YAG laser was used as the source of light. The single-element ultrasound transducer (V309 Panametrics) with a central frequency of 5 MHz and a diameter of 12.7 mm was used to receive the ultrasound signals. At each signal acquisition position, the photoacoustic signals were first amplified by a pulse amplifier, then recorded with an oscilloscope (MSO4000B, Tektronix), and finally input into a personal computer for signal processing and image reconstruction.

The imaged phantom we used in the experiment is made by gelatin cylinder. The agar phantom was made by mixing 1% lipid, 6% gelatin, and 93% water to simulate biological tissue.  Figure 9(b) is the photograph of the phantom. The diameter of the phantom is 20 mm. One graphite rod with a diameter of 0.5 mm and two hairs of lengths of 4 mm were embedded as the optical absorbers. In the phantom experiment, 60-view data are selected for reconstruction.

In the experiment, 40-view and 80-view signals that are uniformly distributed at a 360° curve are collected to reconstruct images.  Figure 10 displays the images that were reconstructed from the sampling data sets utilizing TVAL3, L1magic, NESTA, and TwIST, respectively. The second row of Figure 10 is reconstructed from 80-view data. When the sampling signals is sufficient, the TVAL3, L1magic, and NESTA methods can construct good-quality images, and the TVAL3 method has the best reconstructed image quality. However, the quality of the reconstructed image with the TwIST method is still relatively poor. When we reconstruct the image with 40-view data (first row of Figure 8), the reconstructions are seriously affected and there are more noise in the images. Only the image reconstructed by the TVAL3 algorithm is relatively clear, while the noises in the reconstructions of the L1magic and NESTA methods affect the identification of the boundary of the phantom.

## 4. Conclusion

In this paper, we have tested and evaluated four reconstruction algorithms (TVAL3, L1magic, NESTA and TwIST) for PAI images with sparsely sampled data. The numerical simulations demonstrate that the TVAL3 method has the most accurate reconstruction performance under sparse sampling while the TwIST method has the worst detail reconstruction ability. In terms of CPU time, the TwIST method needs the least amount of CPU time, and the L1magic method requires the longest CPU time. In terms of the reconstructed image quality, the TVAL3 algorithm has better accuracy and antinoise ability than the other three algorithms. In conclusion, the TVAL3 algorithm has the best image quality and requires less CPU time, which provides a good balance between the accuracy and efficiency of the reconstruction. We believe that the findings of this research will provide insight for the development and application of algorithms in the field of PAI.

## Figures and Tables

**Figure 1:** The NCAT phantom and blood vessel phantom employed in comparisons.

**Figure 2:** Reconstruction results of the NCAT phantom. The first to the third rows are the reconstruction images with 20-view, 30-view, and 40-view that are uniformly distributed at a 360° curve. The first to the fourth columns show the results of TVAL3, L1magic, NESTA, and TwIST individually.

**Figure 3:** Gray curves along the middle extraction line in Figure 1(a). The gray curves are reconstructed with these four algorithms from 20-view, 30-view, and 40-view signals for the NCAT phantom.

**Figure 4:** Reconstruction results of the blood vessel phantom. The first to the third rows are the reconstruction images with 20-view, 30-view, and 40-view that are uniformly distributed at a 360° curve. The first to the fourth columns show the results of TVAL3, L1magic, NESTA, and TwIST individually.

**Figure 5:** Gray curves along the middle extraction line in Figure 1(b). The gray curves are reconstructed with these four algorithms from 20-view, 30-view, and 40-view signals for the NCAT phantom.

**Figure 6:** Comparison of the SNR and NMAE values from the reconstruction results of the NCAT phantom with different numbers of sampling points. The first to the fourth columns show the results of noisy observation with *SNR* = 40, 30, 20, and 10 dB, respectively.

**Figure 7:** Comparison of the SNR and NMAE values from the reconstruction results of the blood vessel phantom with different numbers of sampling points. The first to the fourth columns show the results of noisy observation with SNR = 40, 30, 20, and 10 dB, respectively.

**Figure 8:** The histogram of the influence of changing variance of Gaussian noise distribution on the TVAL3 method.

**Figure 9:** (a) The PAI experimental system. (b) The cross-section of a cylinder of a carbon absorption sample.

**Figure 10:** The first and second rows are the reconstruction images of the carbon absorption sample from 40-view and 80-view experimental data. The first to the fourth columns show the results of TVAL3, L1magic, NESTA, and TwIST individually.

**Table 1:** Numerical results of the NCAT phantom with different sampling positions.

Experimental	CPU time (seconds)				SNR (dB)				NMAE			
Positions	TVAL3	L1magic	NESTA	TwIST	TVAL3	L1magic	NESTA	TwIST	TVAL3	L1magic	NESTA	TwIST
5	2.69	202.84	1.64	1.06	10.01	2.28	6.5	0.76	26.78	65.22	40.13	77.69
10	4.29	298.61	2.23	1.98	15.03	6.3	8.42	0.72	15.02	41.05	32.16	78.04
15	6.16	442.24	2.81	1.8	20.35	8.44	9.85	1.4	8.14	32.09	27.29	72.14
20	8.11	470.25	3.47	3.01	25.28	10.56	10.95	1.93	4.62	25.14	24.04	67.93
25	9.02	425.4	3.89	4.05	29.79	12.27	11.83	2.74	2.75	20.65	21.71	61.83
30	9.93	474.47	4.33	3.13	33.3	13.3	12.31	4.19	1.83	18.34	20.56	52.33
35	10.59	446.89	4.78	3.71	37.09	14.55	13.11	6.15	1.18	15.87	18.74	41.77
40	10.93	444.98	5.06	4.78	40.83	15.62	13.86	9.3	0.77	14.04	17.18	29.06
45	10.94	532.55	5.44	2.2	42.53	17.29	14.33	7.16	0.63	11.58	16.28	37.17
50	10.99	509.73	5.89	3.92	45.71	18.27	15.06	14.36	0.44	10.35	14.98	16.23
55	12.16	474.01	6.27	3.61	48.34	19.4	15.7	18.33	0.32	9.09	13.91	10.28
60	11.8	559.14	6.81	4.33	51.05	20.87	16.3	27.72	0.24	7.67	12.98	3.49
Average	8.97	440.09	4.39	3.13	33.28	13.26	12.35	7.9	5.23	22.59	21.66	45.66

**Table 2:** Numerical results of the blood vessel phantom with different sampling positions.

Experimental	CPU time (seconds)				SNR (dB)				NMAE			
Positions	TVAL3	L1magic	NESTA	TwIST	TVAL3	L1magic	NESTA	TwIST	TVAL3	L1magic	NESTA	TwIST
5	2.68	258.02	1.5	0.29	2.58	0.1	1.59	0.05	71.86	95.62	80.54	97.03
10	4.3	280.44	1.8	0.56	6.07	0.89	2.38	0.36	48.09	87.3	73.56	93.73
15	6.31	338.66	2.24	0.82	9.97	1.98	2.99	0.8	30.71	77.04	68.55	89.99
20	8.22	366.16	2.59	1.19	15.55	2.54	3.69	1.2	16.14	72.26	63.28	84.25
25	10	411.43	2.92	1.48	22.63	3.66	4.38	2.98	7.15	63.51	58.41	68.62
30	11.88	467.69	3.4	1.65	34.49	4.82	4.73	5.08	1.83	55.53	56.12	53.94
35	13.17	481.37	3.87	1.94	42.76	6.31	5.48	10.95	0.7	46.8	51.46	27.42
40	11.91	619.74	4.59	2.53	48.43	7.65	6.36	19.28	0.37	40.11	46.51	10.51
45	12.22	524.17	4.77	2.13	51.61	9.18	6.71	20.4	0.25	33.64	44.71	9.24
50	12.09	672.54	5.39	2.18	54.11	10.8	7.4	23.03	0.19	27.92	41.27	6.83
55	11.3	551.73	5.49	2.81	55.39	12.57	8.21	25.27	0.16	22.76	37.6	5.27
60	12.29	626.07	5.95	2.65	57.93	14.47	8.79	26.56	0.12	18.29	35.19	4.54
Average	9.7	466.5	3.71	1.69	33.46	6.25	5.23	11.33	14.8	53.4	54.77	45.95

## Data Availability

The data that support the findings of this study are available from the corresponding author upon reasonable request.
